# Nucleus pulposus cell apoptosis is attenuated by CDMP-2 through regulating oxidative damage under the hyperosmotic environment

This article has been retracted.

**DOI:** 10.1042/BSR20181176

**Published:** 2018-10-10

**Authors:** Shouguo Jiao, Jingxiang Li, Binbin Liu, Ming Yang, Jiangli Xiu, Daokui Qu

**Affiliations:** 1 Department of Orthopedics, Yantai Yeda Hospital, Yantai 264006, Shandong, China; 2 Department of Traumatic Orthopedics, The Central Hospital of Zaozhuang Mining Group, Zaozhuang 277000, Shandong, China; 3 Department of Operating Room, Yantai Yeda Hospital, Yantai 264006, Shandong, China

**Keywords:** apoptosis, CDMP-2, intervertebral disc degeneration, nucleus pulposus, osmolarity

## Abstract

Disc nucleus pulposus (NP) cell experiences periodic osmolarity alterations during daily activities, which has been proved to affect cell biology *in vitro*. The present study was aimed to investigate the effects of cartilage-derived morphogenetic protein-2 (CDMP-2) on NP cell apoptosis under the hyperosmolarity culture and the potential mechanism. Isolated rat NP cells were cultured in the *in situ*-osmolarity medium or hyperosmolarity medium for 3 days. CDMP-2 was added into the hyperosmolarity medium to investigate its effects on NP cell apoptosis. Cell apoptosis rate, caspase-3 activity, gene expression of Bcl-2, Bax, and caspase-3, and protein expression of Bcl-2, Bax, and cleaved caspase-3 were analyzed to evaluate NP cell apoptosis. Additionally, the intracellular reactive oxygen species (ROS) and the total superoxide dismutase (SOD) activity were analyzed to investigate the potential role of oxidative damage in this process. In the hyperosmolarity culture, NP cells showed a significantly increased cell apoptosis rate and caspase-3 activity, an up-regulated expression of Bax and caspase-3/cleaved-caspase-3 and a down-regulated expression of Bcl-2. However, CDMP-2 partly inhibited these effects of hyperosmolarity culture on NP cells. Additionally, the hyperosmolarity culture significantly increased ROS content and decreased the total SOD activity compared with the *in situ*-osmolarity culture, whereas exogenous CDMP-2 partly decreased the ROS content and increased the total SOD activity in the hyperosmolarity culture. In conclusion, CDMP-2 is effective in attenuating hyperosmolarity environment-induced NP cell apoptosis, and this process may be mediated through inhibiting oxidative stress damage. The present study indicates that CDMP-2 may be helpful to retard hyperosmolarity niche-mediated disc degeneration.

## Introduction

Low back pain is the most common physical problem in the orthopedic outpatients [1,2]. It causes a heavy economic burden to family and seriously affects the patient’s daily living. According to previous researches and findings, intervertebral disc degeneration is regarded as the main contributor to low back pain [3,4]. To elucidate the pathogenesis of disc degeneration, increasing evidence have indicated that disc cell apoptosis is responsible for disc degeneration [5–7].

The intervertebral disc consists of the annulus fibrosus (AF), nucleus pulposus (NP), and cartilage endplates (CEPs) [8]. The central gelatinous NP plays an important role in relieving stress and maintaining disc function by distributing the hydraulic pressure evenly to the adjacent AF and CEPs [9]. During disc degeneration, the NP tissue first exhibits degenerative changes, including the decrease in cellular density and matrix production [10]. *In vivo*, the disc NP cells reside in an environment of hyperosmolarity [11,12]. When the discs are subjected to the mechanical compression, the *in situ* osmolarity within the NP region further increased due to the water exclusion from the NP region. Several studies have reported that increased mechanical load promotes disc NP cell apoptosis [13–18]. Because the osmolarity alteration is the secondary change of mechanical compression, several research teams have investigated the effects of osmolarity on NP cell biology. Importantly, these studies have verified that hyperosmolarity induces disc NP cell apoptosis [19–21].

Currently, the existing therapies for disc degeneration are mainly targetted to pain symptoms rather than the underlying pathogenesis. According to the previous studies, it has been established that disc degeneration is a cell-mediated process originating from the disc NP tissue [22]. Therefore, lots of novel biological approaches are being developed to retard disc degeneration by restoring disc matrix or attenuating matrix degradation [23,24]. However, keeping sufficient cell number within the disc tissue is a key precondition for the efficacy of this type of therapies [23]. Because the cellular loss is an obvious and important feature during disc degeneration, the maintenance of adequate cell number within the disc tissue is implicated for the biological treatments of disc degeneration.

Cartilage-derived morphogenetic protein-2 (CDMP-2) is an endogenous growth factor belonging to the BMP family and participates in regulating chondrocyte’s biology [25,26]. Previous studies have demonstrated that CDMP-2 is down-regulated in the osteoarthritic human articular chondrocytes and is able to enhance cartilaginous matrix synthesis [27,28]. Importantly, a previous study has indicated that intradiscal CDMP-2 injection restored NP matrix content and tissue hydration compared with the control discs in the annular injury-induced ovine disc degeneration model [29]. In light of the disc NP tissue is similar to a cartilaginous tissue in some aspects; we deduced that CDMP-2 may also be helpful to maintain the healthy disc biology. In the present study, we mainly aimed to investigate the effects of CDMP-2 on the NP cell apoptosis and the potential mechanism under hyperosmolarity.

## Materials and methods

### NP cell isolation and amplification

Rat NP cells were isolated from 23 Sprague–Dawley rats (male, 7–8 weeks old) according to a previous method [30]. Briefly, after NP tissue samples were separated, NP cells were isolated by digestion with 0.1% collagenase type II (Sigma–Aldrich, U.S.A.) for 4–6 h. All experimental rats were used according to the guidelines of the Ethics Committee at Yantai Yeda Hospital [YD (LU) 2014-0020]. The isolated NP cells were cultured in standard DMEM/F12 culture medium containing 10% FBS (Gibco, U.S.A.) in 95% humidity, 21% O_2_, and 5% CO_2_ at 37°C. When they were grown to 80% confluence, NP cells were subcultured. The passage 2 NP cells were seeded in the six-well culture plate and used for every test in the present study.

### NP cell culture under hyperosmolarity

The control NP cells were cultured in the *in situ*-osmolarity (450 mOsm/kg) medium, whereas the experimental NP cells were cultured in the hyperosmolarity (550 mOsm/kg) medium for 3 days. Because the NP tissue osmolarity alters between 400 and 450 mOsm/kg [31], the *in situ*-osmolarity value was designed as 450 mOsm/kg, whereas the hyperosmolarity value was designed as 550 mOsm/kg. To study the effects of CDMP-2 on NP cell apoptosis under hyperosmolarity, CDMP-2 (100 ng/ml, PeproTech, Rocky Hill, NJ, U.S.A.) was added along with the hyperosmolarity culture medium. Here, the osmolarity value was adjusted by sucrase and verified by a freezing point osmotic pressure instrument (FM-8P, Bejing Xin Xiao Tengda Instrument Equipment Co., Ltd, China). All NP cells were cultured in the different types of medium for 3 days before each test.

### Flow cytometry assay

After culture, NP cell apoptosis ratio was evaluated by the method of annexin V-FITC/PI staining (Beyotime, China) according to the instructive steps. Briefly, the cultured NP cells were washed with phosphate buffer solution (PBS) for two times. Then, they were incubated with 0.25% trypsin (Gibco, U.S.A.) and collected by centrifugation (1000 ***g***, 4°C) for 3 min. Thereafter, 1 × 10^5^ NP cells in each group were incubated with 195 μl Annexin V-FITC combination buffer, 5 μl Annexin V-FITC solution, and 10 μl PI solution for 20 min in the dark environment. Then, the processed NP cells were subjected to a flow cytometry machine and apoptotic NP cells, including the early and terminal apoptotic cells were calculated.

### Measurement of caspase-3 activity

Briefly, after NP cells were incubated with different types of osmolarity medium, they were lysed by the lysis solution. Then, the protein supernatant was collected by centrifugation and the reactive system was developed based on the manufacturer’s instructions (caspase-3 Activity Detection Kit, Beyotime, China). Finally, the optical density (OD) at a wavelength of 405 nm was measured and the caspase-3 activity was calculated according to the standard curve.

### Measurement of total superoxide dismutase activity

Briefly, after NP cells were incubated with different types of osmolarity medium, they were incubated with the lysis buffer and the supernatant was collected by centrifugation. Then, the superoxide dismutase (SOD) activity was measured using a Total SOD Assay Kit (Beyotime, China). Finally, SOD activity was expressed as U/mg protein.

### Measurement of reactive oxygen species content

Reactive oxygen species (ROS) content was analyzed using a ROS Assay Kit according to the manufacturer’s instructions (Beyotime, China). Briefly, after NP cells were incubated with different types of osmolarity medium, they were stained with 10 μM DCFH-DA solution for 20 min at 37°C in the dark environment. Then, the relative fluorescence units (RFU) at an excitation/emission wavelength of 488/525 nm was measured using an automatic microplate reader (Thermo Fisher Scientific, U.S.A.).

### Real-time PCR

After NP cells were incubated with different types of osmolarity medium, total RNA of NP cells was extracted using 1 ml of TRIzol reagent (Invitrogen, U.S.A.) and reverse-transcribed to synthesize cDNA templates using a Reverse Transcription Kit (TIANGEN, China) according to the manufacturer’s instructions. The primers of the target genes were shown in the Table 1. Then, the real-time PCR assay was performed on a reaction system containing cDNA templates, primers, and SYBR Green mix (Dongsheng Biotech, China). The PCR procedure was processed according to the follow conditions: 5 min at 95°C, followed by 30 amplification cycles of 10 s at 95°C, 8 s at 57°C, and 8 s at 72°C. The relative gene expression level was calculated according to the method of 2^−ΔΔ*C*^_T_ and normalized to the housekeeping gene *β-actin*.

**Table 1:** Primers of target genes

Gene	Forward (5′–3′)	Reverse (5′–3′)
*β-actin*	CCGCGAGTACAACCTTCTTG	TGACCCATACCCACCATCAC
*Bcl-2*	GGGGCTACGAGTGGGATACT	GACGGTAGCGACGAGAGAAG
*Bax*	GGCGAATTGGCGATGAACTG	CCCAGTTGAAGTTGCCGTCT
*Caspase-3*	GGAGCTTGGAACGCGAAGAA	ACACAAGCCCATTTCAGGGT

### Western blot assay

After NP cells were incubated with different types of osmolarity medium, they were incubated by lysis buffer (Beyotime, China) and total protein was extracted according to the instructions. Protein concentration in each group was measured using a BCA protein assay kit (Beyotime, China). Then, equal amount of protein samples in each group were separated via SDS/PAGE and transferred on to the PVDF membranes. After the PVDF membranes were blocked with 5% BSA for 1 h at room temperature, they were incubated overnight at 4°C with primary antibodies (anti-β-actin: Abcam, ab8226, anti-cleaved caspase-3: Cell Signaling Technology, #9661; anti-Bcl-2: Proteintech, 12789-1-AP; anti-Bax: Proteintech, 50599-2-Ig; all were diluted at 1:1000). On the following day, the PVDF membranes were incubated for 2 h at room temperature with the horseradish peroxidase–conjugated secondary antibodies (diluted at 1:200, Beyotime, China). Thereafter, protein bands were developed using the ECL Plus (Thermo, U.S.A.) according to the manufacturer’s instructions. After gray value analysis using the Quantity One software (Bio-Rad, U.S.A.), protein expression of one target molecule was expressed as the ratio of its gray value to that of β-actin.

### Statistical analysis

All numerical data in the present study are showed as the means ± S.E.M. of three independent replicates. The data were analyzed using the SPSS 19.0 software with the method of one-way ANOVA followed by the LSD post test to compare the difference between two groups. A *P*-value <0.05 indicated a statistical significance.

## Results

### NP cell apoptosis ratio

Results showed that NP cell apoptosis rate in the hyperosmolarity culture group was significantly increased compared with the *in situ*-osmolarity culture group, whereas CDMP-2 partly decreased NP cell apoptosis rate in the hyperosmolarity culture group (Figure 1).

**Figure 1:** Analysis of NP cell apoptosis ratio Data are expressed as mean ± S.D., *n*=3. *: Indicates a significant difference (*P*<0.05) between two groups.

### Caspase-3 activity

Results showed that caspase-3 activity in the hyperosmolarity culture group was significantly increased compared with the *in situ*-osmolarity culture group, and CDMP-2 partly decreased caspase-3 activity in the hyperosmolarity culture group (Figure 2).

**Figure 2:** Analysis of caspase-3 activity of NP cells Data are expressed as mean ± S.D., *n*=3. *: Indicates a significant difference (*P*<0.05) between two groups.

### Gene expression analysis

Hyperosmolarity culture significantly down-regulated gene expression of anti-apoptosis molecule (Bcl-2) compared with the *in situ*-osmolarity culture group, whereas CDMP-2 partly increased *Bcl-2* mRNA expression in the hyperosmolarity culture group. However, hyperosmolarity culture significantly up-regulated gene expression of pro-apoptosis molecules (Bax and caspase-3) compared with the *in situ*-osmolarity culture group, whereas CDMP-2 partly decreased mRNA expression of Bax and caspase-3 in the hyperosmolarity culture group (Figure 3).

**Figure 3:** Analysis of mRNA expression of apoptosis-related molecules (Bcl-2, Bax, and caspase-3) in NP cells Data are expressed as mean ± S.D., *n*=3. *: Indicates a significant difference (*P*<0.05) between two groups.

### Protein expression analysis

Results showed that hyperosmolarity culture significantly increased protein expression of cleaved-caspase-3 and Bax compared with the *in situ*-osmolarity culture group, and addition of CDMP-2 partly decreased their expression in the hyperosmolarity culture. Inversely, protein expression of Bcl-2 showed an opposite pattern compared with that of cleaved caspase-3 and Bax amongst these groups (Figure 4).

**Figure 4:** Analysis of protein expression of apoptosis-related molecules (Bcl-2, Bax, and cleaved caspase-3) in NP cells Data are expressed as mean ± S.D., *n*=3. *: Indicates a significant difference (*P*<0.05) between two groups.

### ROS content analysis

Results showed that ROS content in the hyperosmolarity culture group was significantly increased compared with the *in situ*-osmolarity culture group, whereas CDMP-2 partly decreased ROS content in the hyperosmolarity culture group (Figure 5).

**Figure 5:** Measurement of intracellular ROS content in NP cells Data are expressed as mean ± S.D., *n*=3. *: Indicates a significant difference (*P*<0.05) between two groups.

### SOD activity analysis

Results showed that the total SOD activity in the hyperosmolarity culture group was significantly decreased compared with the *in situ*-osmolarity culture group, whereas CDMP-2 partly increased the total SOD activity in the hyperosmolarity culture group (Figure 6).

**Figure 6:** Measurement of total SOD activity in NP cells Data are expressed as mean ± S.D., *n*=3. *: Indicates a significant difference (*P*<0.05) between two groups.

## Discussion

Disc degeneration is an important contributor to low back pain [3]. Currently, its pathogenesis is unclear and no effective treatments are developed to biologically regenerate the degenerative disc [9]. Disc cell apoptosis is an underlying mechanism of disc degeneration [5,6]. Though several previous studies have demonstrated that hyperosmolarity culture promotes disc NP cell apoptosis [19–21], the potential mechanism and the prevention strategies are not better understood. The present study confirmed that hyperosmolarity culture promoted NP cell apoptosis and first reported that CDMP-2 attenuated hyperosmolarity culture-induced NP cell apoptosis through alleviating the oxidative stress injury. The present study shed a new light on the protective effects of CDMP-2 against NP cell apoptosis caused by the hyperosmolarity environment.

Previously, disc NP cell apoptosis has attracted lots of attention around the world. Gruber and Hanley [32] first identified the apoptotic disc cells in the degenerative disc tissue. Subsequently, Rannou et al. [33] demonstrated a positive relationship between NP cell apoptosis and disc degeneration in humans. Because cellular loss from excessive disc cell apoptosis contributes to the decrease in extracellular matrix content, and thus plays an important role in the process of IVD degeneration [5,6], inhibition of disc cell apoptosis may be a promising strategy to retard disc degeneration. Previously, gene technologies and caspase inhibitors have been used to inhibit disc cell apoptosis and exhibited promising results *in vivo* and *in vitro* [34–37].

Under the physiological conditions, the disc is intermittently subjected to various mechanical stimuli, which induces fluid inflow and outflow of disc tissue [38,39]. The fluid volume of the disc tissue directly causes the alteration of the *in situ* osmolarity. Previously, several studies have demonstrated that both the high mechanical compression and hyperosmolarity culture promoted disc NP cell apoptosis [13,15–21]. In the present study, we found that NP cells in the hyperosmolarity culture showed an increased apoptosis ratio and caspase-3 activity, an up-regulated expression of pro-apoptosis molecules (Bax and caspase-3/cleaved caspase-3), but a decreased expression of anti-apoptosis molecule (Bcl-2) compared with the NP cells in the *in situ*-osmolarity culture. These results confirm again that hyperosmolarity promotes the process of NP cell apoptosis. However, our results also showed that CDMP-2 partly decreased apoptosis ratio and caspase-3 activity, down-regulated expression of pro-apoptosis molecules (Bax and caspase-3/cleaved caspase-3), and increased expression of anti-apoptosis molecule (Bcl-2) in the hyperosmolarity culture, indicating that CDMP-2 is able to inhibit hyperosmolarity culture-induced NP cell apoptosis. Previously, Le Maitre et al. [40] identified that CDMP-2 expression was decreased in the NP cells from the degenerative discs and indicated that CDMP-2 was able to promote matrix synthesis of NP cells. This is indirectly in line with us and suggests again that CDMP-2 may be helpful to retard disc degeneration.

Oxidative stress injury is a classical pathological process in many diseases, such as cardiovascular disease, diabetes, and osteoarthritis [41–43]. Increasing studies have indicated that initiation and aggravation of disc degeneration are closely associated with oxidative stress damage [44–46]. As an important initiator of disc degeneration, mechanical load also increases generation of the intracellular ROS, and causes oxidative damage [47–51]. As the secondary event of mechanical compression, the hyperosmolarity environment also causes oxidative damage in corneal epithelial cells [52]. In the present study, we found that hyperosmolarity culture increased ROS generation and decreased the total SOD activity compared with the *in situ*-osmolarity culture, whereas CDMP-2 partly decreased ROS generation and increased the total SOD activity in the hyperosmolarity culture. In light of the alteration of NP cell apoptosis before and after addition of CDMP-2, these results indicate that CDMP-2 may inhibit NP cell apoptosis under the hyperosmolarity environment through attenuating the oxidative damage.

However, our study also has several limitations. First, the NP cells were isolated from the rat NP tissue in the present study. As we know, the rat NP tissue contains lots of notochordal cells, whereas the adult human disc NP tissue almost contains no notochordal cells. Hence, the existence of notochordal cells may cause interference to the present results. Second, the disc contains three structurally connected parts: NP, AF, and CEPs. The present study only performed an *in vitro* study in the NP cell culture. To verify the conclusion of the present study, a disc organ culture study may be an important supplement.

## Conclusion

In a word, we observed the protective effects of CDMP-2 against hyperosmolarity environment-caused disc NP cell apoptosis and investigated the underlying mechanism. Our results demonstrated that CDMP-2 attenuated NP cell apoptosis under hyperosmolarity culture, and that this process may be mediated through inhibiting the oxidative stress injury. The present study provides protective new knowledge about the effects of CDMP-2 against NP cell apoptosis caused by the hyperosmolarity environment and is helpful to better understand disc degeneration.

## Abbreviations

AF: annulus fibrosus
BMP: bone morphogenetic protein
CDMP-2: cartilage-derived morphogenetic protein-2
CEP: cartilage endplate
DCFH-DA: 2′,7′-dichlorodihydrofluorescein diacetate
DMEM/F12: Dulbecco’s modified Eagle medium/nutrient mixture F-12
IVD: intervertebral disc
LSD: least significant difference
NP: nucleus pulposus
PI: propidium iodide
ROS: reactive oxygen species
SOD: superoxide dismutase
